The article "A highly significant association between Cathepsin S gene polymorphisms rs12068264 and chronic obstructive pulmonary disease susceptibility in Han Chinese population" was published in 2018. Journal: Biosci Rep.

# A highly significant association between Cathepsin S gene polymorphisms rs12068264 and chronic obstructive pulmonary disease susceptibility in Han Chinese population

**DOI:** 10.1042/BSR20180410

**Published:** 2018-07-18

**Authors:** Sheng-lan Gao, Ya-hong Wang, Chun-yan Li, La-wei Yang, Bao-an Zou, Zu-guang Chen, Wei-min Yao, Ze-qing Song, Jun-fen Cheng, Zi-ying Lin, Gang Liu

**Affiliations:** 1 Clinical Research Center, Affiliated Hospital of Guangdong Medical University, Zhanjiang 524001, China; 2 Department of Respiratory Medicine, Affiliated Hospital of Guangdong Medical University, Zhanjiang 524001, China; 3 Institute of Respiratory Disease, The Second People’s Hospital of Zhanjiang, Zhanjiang 524003, China

**Keywords:** CTSS, chronic obstructive pulmonary disease, Chinese population, genetic polymorphism, SIRT1

## Abstract

Cathepsin S (CTSS) and Sirtuin-1 (SIRT1) played crucial roles in the pathogenesis of chronic obstructive pulmonary disease (COPD). However, the associations between the polymorphisms of CTSS as well as SIRT1 and COPD in Asian population remain elusive. In the present study, one single nucleotide polymorphism (SNP) in rs12068264 was discovered (in 385 individuals) to be associated with the susceptibility of COPD in a Chinese Han population. The genotyping was performed using improved multiplex ligase detection reaction (iMLDR) technique. Subjects with T allele of rs12068264 in CTSS gene had an increased risk of COPD (T compared with C: odds ratio (OR) = 1.351, 95% confidence interval (95% CI): 1.008–1.811, *P*=0.044) compared with C allele. Subjects with TT genotype at rs12068264 had a higher risk of COPD in a recessive model (TT compared with TC + CC: OR = 2.30, 95% CI: 1.06–4.989, *P*=0.035). Compared with the C variant of rs12068264, the homozygous carriers of the TT genotype had higher procalcitonin (PCT) levels. Finally, haplotype analysis demonstrated that the SNPs in the *CTSS* and *SIRT1* gene had no statistical differences between patients with COPD and the controls. In conclusion, the genetic polymorphisms of CTSS were associated with the susceptibility of COPD in a Chinese Han population, which may be helpful in understanding genetic mechanisms underlying the pathogenesis of COPD.

## Introduction

Chronic obstructive pulmonary disease (COPD) is a major cause of deaths worldwide and is characterized by an irreversible progressive decline in lung function and chronic inflammatory response [1]. The prevalence is approximately 10% in the elderly and this disease is expected to become the third leading cause of deaths by 2030 in the world [2]. COPD is regarded as a systemic disease. Numerous studies demonstrated that oxidative stress, protease–antiprotease imbalance, as well as inflammation played important roles in COPD pathogenesis [3–5]. It is well reported that long-term exposure to cigarette smoke, a predominant risk stimuli for COPD development, leads to cellular oxidative stress and inflammatory response in the airways as well as lungs [3]. Interestingly, there are only 15–20% of smokers reaching COPD, suggesting that genetic factors are implicated in the pathogenesis of the disorder except for environmental factors [6]. The molecular mechanisms underlying COPD pathogenesis are complex and it is very important to identify the genetic susceptibility factor of the development of COPD for early prevention, early detection, and the early treatment of this disease.

The article "A highly significant association between Cathepsin S gene polymorphisms rs12068264 and chronic obstructive pulmonary disease susceptibility in Han Chinese population" was published in 2018. Journal: Biosci Rep.

Increasing evidence suggested that a variety of factors including imbalance of proteases exert a vital role in the development and progression of COPD [4,7,8]. Proteases are able to cleave proteins into smaller fragments, which have regulatory roles in many pathological process such as apoptosis, oxidative stress, and inflammatory response [7]. Therefore, dysregulated proteases are involved in the pathogenesis of various diseases including COPD. Proteinases like neutrophil elastase, matrix metalloproteases, and cysteine proteases are closely associated with development of emphysema and destruction of airways in COPD [9].

Cathepsin S (CTSS) is a cysteine proteinase of the papain superfamily, which is mainly expressed in professional antigen-presenting cells related to COPD-like macrophages, microglia, B lymphocytes, as well as dendritic cells [10,11]. This enzyme plays a crucial action in assembling MHC class II–Ag complexes and promotes antigen processing and presentation and subsequently induces the activation of CD4+ T cells [12]. CTSS levels were elevated in bronchoalveolar lavage fluid and plasma of COPD patients compared with the healthy volunteers [13,14]. Moreover, CTSS is implicated in pathogenesis of alveolar remodeling and pulmonary emphysema in interferon-γ-treated mouse [15,16]. Collectively, CTSS plays an influential role in the pathogenesis of COPD.

Sirtuin-1 (SIRT1) is the best characterized member of silent information regulator (Sir2) family in mammals and is an NAD-dependent protein deacetylase [16]. This enzyme controls numerous cellular responses involved in regulating homeostasis [17] and it is demonstrated to have inhibitory roles in ageing and inflammation [18–20]. SIRT1 is reported to decrease in lungs of COPD patients, the well-known ageing-related and inflammation-associated diseases [1,21], initially reported by Rajendrasozhan et al. [20]. In addition, through deacetylating multiple substrate proteins like Forkhead box O proteins (FOXOs), p53, and nuclear factor-κB, SIRT1 exerts an important role in the cellular responses to oxidative stress, cellular senescence, and modulation of inflammation in COPD [22]. These observations indicated that SIRT1 has important functions in the progression of COPD.

The article "A highly significant association between Cathepsin S gene polymorphisms rs12068264 and chronic obstructive pulmonary disease susceptibility in Han Chinese population" was published in 2018. Journal: Biosci Rep.

COPD is a complicated disease and is at least partly determined by gene(s). Increasing evidence suggested that single nucleotide polymorphisms (SNP) distribution of genes implicated in COPD such as *IL-13, FAM13A*, and *VEGFA* genes play key roles in the COPD development [23–25]. However, the SNP-caused effects of many genes involved in COPD susceptibility and progression remain largely unknown. Therefore, the purpose of the present study was to investigate the associations between CTSS and SIRT1 SNPs and the susceptibility of COPD in a Chinese population.

## Materials and methods

### Study subjects

Cases (182) and controls (203) were selected as our research objects in the hospital-based case–control study. The control samples were obtained from medical examination center of Affiliated Hospital of Guangdong Medical University and cases were collected from Affiliated Hospital of Guangdong Medical University as well as The Second People’s Hospital of Zhanjiang from June 2015 to June 2017. All the cases were diagnosed newly with forced expiratory volume in 1 s (FEV1) for the reason that FEV1 over forced vital capacity (FEV1/FVC) < 0.7 has become the gold criteria for diagnosing COPD [26,27]. The controls who were free from a history of cancer and respiratory diseases were randomly selected in the same hospital during the same period. The present study was approved by the institutional review board of Guangdong Medical University.

### Candidate SNP selection and genotyping

The characteristics of two SNPs (rs12068264 and rs11576175) of *CTSS* gene and three SNPs (rs2273773, rs16924934, and rs3818291) of *SIRT1* gene selected for the test are shown in Table 1. Whole blood samples (5 ml) were collected from each control and COPD patients during a laboratory examination. Genomic DNA was extracted from whole blood using a commercially available DNA isolation kit (Tiangen Biochemical Technology, Beijing, China) following the manufacturer’s protocol. SNPs were used based on their frequencies and positions, as well as their relationship with infectious diseases documented previously. SNP genotyping was performed using an improved multiplex ligation detection reaction (iMLDR) technique (Genesky Biotechnologies Inc., Shanghai, China).

**Table 1:** Basic SNP information of *CTSS* and *SIRT1* genes examined in the study

Gene	SNP ID	Chr.	Chr. position	SNP property	Alleles	Allele 1	Allele 2
*CTSS*	rs12068264	1	150727329	intron3	C/T	C	T
*CTSS*	rs11576175	1	150727394	intron3	G/A	G	A
*SIRT1*	rs2273773	10	69666598	synon_exon4	C/T	C	T
*SIRT1*	rs16924934	10	69664933	intron3	G/A	G	A
*SIRT1*	rs3818291	10	69672999	intron7	G/A	G	A

Abbreviation: Chr., chromosome.

The article "A highly significant association between Cathepsin S gene polymorphisms rs12068264 and chronic obstructive pulmonary disease susceptibility in Han Chinese population" was published in 2018. Journal: Biosci Rep.

### Statistical analysis

All statistical analyses were two-tailed and conducted with SPSS 18.0. A value of *P*<0.05 was defined as the criterion of statistical significance. Hardy–Weinberg equilibrium (HWE) was tested by a goodness-of-fit χ^2^ test. Student’s *t*test was performed in continued variables and the Pearson’s χ^2^ was performed in categorical variables between cases and controls. The odds ratios (OR) and 95% confidence intervals (95% CI) were calculated to estimate the association between SNP and the risk of COPD by logistic regression analysis after adjustment of age and gender. In addition, the haplotype analysis of CTSS and SIRT1 polymorphisms was determined using the Haploview 4.2 program. Only those haplotypes with frequencies greater than 3% were further analyzed.

## Results

### CTSS and SIRT1 SNPs genotype and allele frequencies

Genotype distributions and allele frequencies of CTSS and SIRT1 SNPs in the COPD group and the control group are listed in Table 2. Genotype distributions of all polymorphisms were found to conform to HWE (*P*>0.05), indicating that our subjects presented the source population well. A statistical difference was observed between the patients with COPD and the controls in the distribution of CTSS rs12068264 genotypes (*P*=0.048). The prevalence of rs12068264 T-allele frequencies in *CTSS* gene was significantly higher in COPD patients than in controls (T compared with C: OR = 1.351, 95% CI: 1.008–1.811, *P*=0.044). In addition, for the other polymorphisms, no significant differences were observed in the genotype and allele frequencies between the COPD patients and the control groups.

**Table 2:** Frequencies of genotype and allele of CTSS and SIRT1 SNPs in the control and COPD groups

SNP	Group	Genotype number			*P*	HWE *P*	Allele freq (%)		*P*	OR (95% CI)
rs12068264		TT	TC	CC			T	C		
	Control	21	96	85	0.048	0.531	34.16%	65.84%	0.044	1.351 (1.008–1.811)
	COPD	35	80	67		0.222	41.21%	58.79%		
rs11576175		AA	AG	GG			A	G		
	Control	10	62	131	0.506	0.512	20.2%	79.8%	0.234	0.801 (0.555–1.155)
	COPD	6	49	126		0.600	16.85%	83.15%		
rs16924934		GG	GA	AA			G	A		
	Control	6	54	143	0.908	0.795	16.26%	83.74%	0.773	1.058 (0.724–1.546)
	COPD	5	52	125		1	17.03%	82.97%		
rs2273773		CC	CT	TT			C	T		
	Control	10	77	116	0.208	0.700	23.89%	76.11%	0.084	1.326 (0.962–1.828)
	COPD	15	77	90		0.860	29.4%	70.6%		
rs3818291		AA	AG	GG			A	G		
	Control	8	55	140	NA	0.340	17.49%	82.51%	0.868	0.969 (0.666–1.409)
	COPD	3	56	123		0.302	17.03%	82.97%		

Abbreviation: Freq, frequency. NA, not available.

The article "A highly significant association between Cathepsin S gene polymorphisms rs12068264 and chronic obstructive pulmonary disease susceptibility in Han Chinese population" was published in 2018. Journal: Biosci Rep.

### Association analysis of CTSS and SIRT1 polymorphisms and risk of COPD in dominant and recessive model

The age and gender analysis showed COPD patients had older age than the controls (71.67 ± 10.43 compared with 55.48 ± 10.62, *P*<0.001) and the COPD cases and control subjects exhibited significant difference in gender (145 males and 37 females compared with 111 males and 92 females, *P*<0.001). Subsequently, to investigate the association between the CTSS and SIRT1 SNPs associated with COPD, we compared the genotype frequencies of every polymorphism between groups under the dominant and recessive genetic models using logistic regression analysis after adjustment for age and sex. For every SNP, if the frequency of one allele was relatively lower than that of another allele, it was defined as minor allele, which was recognized as a risk allele compared with a wild-type allele. As shown in Table 3, the minor allele T at rs12068264 of *CTSS* gene was associated with an increased COPD risk under a recessive model (TT compared with TC + CC: OR = 2.30, 95% CI: 1.06–4.989, *P*=0.035). However, no significant associations were observed between the other SNPs and the risk of COPD in genotype comparisons under different genetic models.

**Table 3:** Logistic regression analysis of CTSS and SIRT1 polymorphisms and risk of COPD in dominant and recessive model

SNP	Group	Dominant		OR (95% CI)*	P*	Recessive		OR (95% CI)*	P*
rs12068264		TT + TC	CC			TT	TC + CC		
	Control	117	85	1.014 (0.596–1.723)	0.960	21	181	2.30 (1.06–4.989)	0.035
	COPD	115	67			35	147		
rs11576175		AA + AG	GG			AA	AG + GG		
	Control	72	131	0.760 (0.435–1.327)	0.334	10	193	0.505 (0.124–2.055)	0.340
	COPD	55	126			6	175		
rs16924934		GG + GA	AA			GG	GA + AA		
	Control	60	143	0.953 (0.545–1.669)	0.867	6	197	0.556 (0.137–2.267)	0.413
	COPD	57	125			5	177		
rs2273773		CC + CT	TT			CC	CT + TT		
	Control	87	116	1.578 (0.935–2.664)	0.088	10	193	1.333 (0.476–3.74)	0.585
	COPD	92	90			15	167		
rs3818291		AA + AG	GG	1.281 (0.731–2.244)	0.387	AA	AG + GG	0.386 (0.072–2.063)	0.266
	Control	63	140			8	195		
	COPD	59	123			3	179		

* OR and *P*-value was adjusted by age and gender.

### Correlation analysis between rs12068264 of *CTSS* gene and clinical characteristics of COPD patients

For further analysis, we also focussed on the description of general clinical characteristics of 132 patients with COPD by genotype and we found that the FEV1/FVC ratio and FEV1/predicted of these COPD subjects were 57.69 ± 14.22, 53.66 ± 22.89, respectively. As shown in Table 4, the homozygous carriers of the TT genotype for the rs12068264 polymorphism was associated with higher levels of procalcitonin (PCT) compared with the presence of the C variant (*P*=0.043). Nevertheless, there were no significant associations of the genotype of rs12068264 with duration of illness, years of smoke, age at onset, gender, and the prevalence of pulmonary heart disease and combined severe pneumonia. Moreover, the association between rs12068264 and the levels of white blood cell (WBC) count, neutrophil granulocyte ratio (N%), C-reactive protein (CRP), FEV1/FVC, FEV1/predicted did not show significance .

The article "A highly significant association between Cathepsin S gene polymorphisms rs12068264 and chronic obstructive pulmonary disease susceptibility in Han Chinese population" was published in 2018. Journal: Biosci Rep.

**Table 4:** Clinical characteristics of the patients with COPD and distribution by genotypes of the rs12068264

Parameters	TT	TC + CC	*P*
Duration of illness (years)	8.871 ± 4.16	9.73 ± 7.12	0.124
Years of smoke (years)	33.37 ± 11.57	33.02 ± 10.97	0.590
WBC (10^9^) count	8.11 ± 3.30	9.70 ± 5.37	0.082
N%	69.49 ± 12.17	71.85 ± 12.67	0.747
PCT (ng/ml)	0.55 ± 0.87	0.28 ± 0.93	0.043
CRP (mg/l)	8.31 ± 4.46	5.57 ± 4.06	0.486
FEV1/FVC	59.4 ± 11.74	57.12 ± 14.96	0.057
FEV1%	53.33 ± 21.54	53.77 ± 23.43	0.508
Age at onset (years)			
<60	3	11	
≥60	30	88	1.000
Gender			
Male	29	78	0.248
Female	4	21	
Pulmonary heart disease			
No	28	86	0.946
Yes	3	12	
Combined severe pneumonia			
No	15	53	0.580
Yes	16	45	

### Haplotype analysis of CTSS and SIRT1 polymorphisms

We also performed a haplotype analysis according to two SNPs of *CTSS* gene (rs12068264 and rs11576175) and three SNPs of *SIRT1* gene (rs16924934, rs2273773, and rs3818291). As shown in Table 5, there are three major haplotypes of CTSS and four major haplotypes of SIRT1 polymorphisms with a frequency above 3% in our samples. Analysis of the haplotype frequencies in both CTSS and SIRT1 polymorphisms showed no significant differences between patients with COPD and the controls.

**Table 5:** Haplotype analysis of CTSS and SIRT1 polymorphisms in COPD and control groups

Haplotype	Freq (case)	Freq (control)	*P*	OR (95% CI)
rs12068264|rs11576175				
CA	0.1685 (61)	0.203 (82)		1.000 (Reference)
TG	0.4088 (149)	0.3416 (139)	0.076	1.441 (0.962–2.158)
CG	0.4227 (154)	0.4554 (185)	0.576	1.119 (0.754–1.660)
rs16924934|rs2273773|rs3818291				
ATA	0.1703 (62)	0.1749 (71)		1.000 (Reference)
ACG	0.294 (107)	0.2389 (97)	0.295	1.263 (0.815–1.957)
GTG	0.1703 (62)	0.1626 (66)	0.768	1.076 (0.662–1.749)
ATG	0.3654 (133)	0.4236 (172)	0.560	0.886 (0.588–1.333)

Haplotype frequency <0.03 in both COPD patients and controls has been dropped.

## Discussion

In the current study, we analyzed the associations between SNPs in the CTSS as well as *SIRT1* gene and COPD risk in Han Chinese population. We found that rs12068264 of CTSS were associated with the risk of COPD in our population. The T allele frequency of rs12068264 was significantly higher in COPD patients than in controls. Furthermore, the rs12068264 was associated with an increased risk of COPD based on recessive models. We also found that the homozygous carriers of the TT genotype showed higher levels of PCT compared with the presence of the C variant in the rs12068264 polymorphism. However, haplotype analysis demonstrated that the haplotypes frequencies of *CTSS* and *SIRT1* genes had no significant differences between the patients with COPD and the control groups.

The article "A highly significant association between Cathepsin S gene polymorphisms rs12068264 and chronic obstructive pulmonary disease susceptibility in Han Chinese population" was published in 2018. Journal: Biosci Rep.

COPD is a major global health concern [28]. The development and progression of COPD is involved in an inflammatory cell profile including macrophages, neutrophils as well as T lymphocytes. It is of great importance for the early diagnosis of COPD due to the remediable characteristics at initial stage of this illness. It is widely accepted that oxidative stress, proteinases, and proinflammatory mediators are involved in the pathogenesis of COPD [3–5]. CTSS and SIRT1 are reported to play crucial roles in COPD development and therefore can serve as potential biomarkers for COPD [14,22,29]. In this study, we evaluated the potential correlations of the two polymorphisms (rs12068264 and rs11576175) of *CTSS* gene and three polymorphisms (rs2273773, rs16924934, and rs3818291) of *SIRT1* gene with COPD in Han Chinese population. A previous study investigated the common functional polymorphisms (rs7534124, rs35989725, rs16827671, and rs34495036) in the 5′-flanking region in the CTSS promoter and found their possible association with pulmonary emphysema in the Japanese population [30]. Our study found that the T allele frequencies at rs12068264 in *CTSS* gene exhibited significantly higher in COPD patients than in controls, indicating that the T allele of rs12068264 may increase the susceptibility of COPD. We also found that there were significant differences in the age and gender in the current case–control hierarchy, therefore we used the prominent phenotypes for the correction of logic regression. Our binary logistic regression analysis verified that the minor allele T at rs12068264 was related to an increase in COPD risk in a recessive model. The statistically significant associated with the SNPs rs12068264 is in the third intron of the *CTSS* gene, which is usually removed during the gene-splicing process. Although they cause no apparent functional change, intronic SNPs may modulate gene function by affecting the regulation of gene expression [31]. Nevertheless, no significant associations were found between the other SNP rs11576175 of *CTSS* gene as well as three SNPs of *SIRT1* gene and COPD risk. A previous study found that AG genotype of rs11576175 had lower risks of metabolic disorders in a Han Chinese population [32]. However, no significant association was observed between SNP rs11576175 of CTSS and risk of COPD in the present study. This inconsistency may contribute to the different roles of SNP rs11576175 in the pathogenesis of the two different disorders. Furthermore, the genotypes frequencies at rs2273773 in SIRT1 had no significant difference between the COPD patients and controls, which is not in line with the previous observation reported by Kalemci et al. [34] that there is a significant difference between TT, TC, and CC genotypes of rs2273773 in the same different group in Muğla province. These conflicting findings may result from some factors, such as clinical heterogeneity, different sample sizes and ethnic differences.

The article "A highly significant association between Cathepsin S gene polymorphisms rs12068264 and chronic obstructive pulmonary disease susceptibility in Han Chinese population" was published in 2018. Journal: Biosci Rep.

Subsequently, we further analyzed the association between general clinical characteristics of COPD patients and rs12068264 polymorphism. The recorded clinical characteristics include duration of illness, years of smoke, age at onset, gender, and the prevalence of pulmonary heart disease and combined severe pneumonia, WBC count, N%, PCT, CRP, FEV1/predicted, FEV1/FVC. Serum PCT is reported to serve as an inflammatory biomarker and become the only increased biomarker in the systemic bacterial infections. Moreover, it is well accepted that the values of serum PCT have been applied to diagnose local bacterial infections with increased sensitivity of detection methods and reduced diagnostic threshold (0.5 µg/l was used as a diagnostic threshold for bacterial infection) [33]. We observed that the TT genotype had significantly higher PCT levels than the C variant. However, there were other infection indexes, such as WBC, CRP, neutrophil proportion etc. The levels of these indexes were similar between TT homozygotes and C allele carriers. This inconsistency might be related to PCT that exhibits higher specificity and sensitivity than other indexes in the diagnosis of bacterial infection. But we cannot rule out the false positive results due to the small sample size in the present study. FEV1/FVC ratio and FEV1/predicted have been commonly used to confirm the diagnosis of COPD. All patients had FEV1 values <80% of predicted, and thus were diagnosed with moderate to severe COPD based on the Global Initiative for Chronic Obstructive Lung Disease [1]. The classification of COPD severity is as following: mild = FEV1 ≥ 80% of predicted; moderate = FEV1 ≥50 to <80% of predicted; severe = FEV1 ≥30 to <50% of predicted; and very severe = FEV1 < 30% of predicted. The value of FEV1/predicted in COPD patients is more than 30% but less than 50% in the present study, which suggest that the COPD patients are in moderate stage. Nevertheless, rs12068264 genotype demonstrated no significant associations with duration of illness, years of smoke, age at onset, gender, and the prevalence of pulmonary heart disease and combined severe pneumonia, WBC count, N%, CRP, FEV1/FVC, and FEV1/predicted. We also carried out the haplotype analysis and the data demonstrated that the haplotype of CTSS and *SIRT1* gene had no significant associations with the risk of COPD progression.

The article "A highly significant association between Cathepsin S gene polymorphisms rs12068264 and chronic obstructive pulmonary disease susceptibility in Han Chinese population" was published in 2018. Journal: Biosci Rep.

Our current study has several limitations. First, this was a hospital-based, case–control study, therefore, a selection bias was unavoidable and the subjects are not fully representative of the general population. Second, the polymorphisms rs12068264 studied, which were in non-functional area, may not offer a comprehensive view of the genetic variability of CTSS. Third, the present study did not investigate whether the SNP regulate *CTSS* gene transcription and protein translation. Fourth, the association between *CTSS* gene rs12068264 polymorphism and clinical symptoms need to be evaluated in future studies. Fifth, the sample size is relatively small. Thus, false positive results could not be excluded. Finally, the mechanism underlying the association between the polymorphisms at rs12068264 of CTSS and the susceptibility of COPD is still unclear. Therefore, further studies with a larger study subjects and functional experiments are required to be performed.

In conclusion, the current study finds that *CTSS* gene rs12068264 polymorphism may be associated with the risk of COPD in a Han Chinese population, this finding is expected to lead to better COPD prevention and therapy strategies.

## Abbreviations

COPD: chronic obstructive pulmonary disease
CRP: C-reactive protein
CTSS: cathepsin S
FEV1: forced expiratory volume in 1 s
FVC: forced vital capacity
HWE: Hardy–Weinberg equilibrium
N%: neutrophil granulocyte ratio
OR: odds ratio
PCT: procalcitonin
SIRT1: Sirtuin-1
SNP: single nucleotide polymorphism
WBC: white blood cell
95% CI: 95% confidence interval
